# Periodontitis Exacerbates Benign Prostatic Hyperplasia through Regulation of Oxidative Stress and Inflammation

This article has been retracted.

**DOI:** 10.1155/2021/2094665

**Published:** 2021-10-18

**Authors:** Cheng Fang, Lan Wu, Ming-Juan Zhao, Tong Deng, Jia-Min Gu, Xing-Pei Guo, Cheng Li, Weiguang Li, Xian-Tao Zeng

**Affiliations:** ^1^Center for Evidence-Based and Translational Medicine, Zhongnan Hospital of Wuhan University, Hubei, Wuhan 430071, China; ^2^Department of Stomatology, Zhongnan Hospital of Wuhan University, Hubei, Wuhan 430071, China; ^3^Department of Urology, Zhongnan Hospital of Wuhan University, Hubei, Wuhan 430071, China; ^4^Institutes of Evidence-Based Medicine and Knowledge Translation, Henan University, Henan, Kaifeng 475000, China

## Abstract

Epidemiological studies demonstrate that men with periodontitis are also susceptible to benign prostatic hyperplasia (BPH) and that periodontal treatment can improve the prostatic symptom. However, molecular links of this relationship are largely unknown. The goal of the current study was to elucidate the effects of experimental periodontitis on the hyperplasia of prostate and whether oxidative stress and inflammation participated in this process. For this purpose, ligature-induced periodontitis, testosterone-induced BPH, and the composite models in rats were established. Four weeks later, all the rats were sacrificed and the following items were measured: alveolar bone loss and histological examination of periodontal tissues were taken to assess the establishment of periodontitis model, prostate index and histological examination of prostate tissues were taken to test the establishment of the BPH model, inflammatory cytokines in plasma were assessed, and Bax/Bcl-2 proteins related to cell apoptosis were analyzed via western blot analysis. To further investigate whether oxidative stress participates in the aggravation of BPH, *in vitro* models were also conducted to measure the production of intracellular reactive oxygen species (ROS) and hydrogen peroxide (H_2_O_2_) concentration. We found that simultaneous periodontitis and BPH synergistically aggravated prostate histological changes, significantly increased Ki67 proliferation, and reduced apoptosis in rat prostate tissues. Also, our results showed that periodontal ligation induced increased Bcl-2 protein expression, whereas Bax expression was decreased in BPH rats than in normal rats. Compared with the control group, periodontitis and BPH both significantly enhanced inflammatory cytokine levels of TNF-*α*, IL-6, IL-1*β*, and CRP. Furthermore, *Porphyromonas gingivalis* lipopolysaccharide induced enhanced generation of intracellular expression of ROS and H_2_O_2_ in BPH-1 cells. Our experimental evidence demonstrated that periodontitis might promote BPH development through regulation of oxidative stress and inflammatory process, thus providing new strategies for prevention and treatment of BPH.

## 1. Introduction

Benign prostatic hyperplasia (BPH) is a common age-related proliferative disease in males, which is characterized by increased number of epithelial and stromal cells in the periurethral area of the prostate [1, 2]. The prevalence of BPH increases from 25% in men aged 40 to 49 years to more than 80% in men aged 70 to 79 years [3]. Periodontitis is another prevalent age-related inflammatory disorder that affects the teeth's supportive tissues, which eventually contributing to tooth loss and systemic inflammation [4]. It is reported that populations aged 55 to 65 years are at the highest risk of developing severe periodontitis [5]. Epidemiological studies have demonstrated that periodontitis obviously raised the risk of BPH after adjusting for confounding factors [6, 7]. In recent years, links between periodontal disease and prostatic disease have gained increasing attention since both diseases share several common risk factors, such as age, metabolic disorders, and psychological factors [8, 9]. We have proposed an oral-prostate axis hypothesis in which periodontitis may act on prostatic disease in a direct way through distant dissemination of oral bacteria (i.e., *Porphyromonas gingivalis*) and/or an indirect way through systemic inflammation; however, the precise mechanisms underlying these relationships are poorly understood [8, 10].

Numerous studies have demonstrated that oxidative stress is involved in the development of both periodontal and prostatic diseases [11, 12]. Oxidative stress is a situation when the oxidation system and antioxidant system is unbalanced with overproduction of reactive oxygen species (ROS) and a comparative deficiency of antioxidants [13]. Excessive accumulation of ROS can induce DNA damage, lipid peroxidation, and protein modification, subsequently causing cellular dysfunction and tissue damage [11, 14]. As one of the main sources of intracellular ROS, hydrogen peroxide (H_2_O_2_) is broadly used as an oxidative stressor in the *in vitro* models. Oxidative stress has been highly associated with the onset of several inflammatory pathologies occurring in elderly people, including periodontitis, osteoporosis, and metabolic disorders [12, 15, 16]. Also, clinical and experimental studies have a confirmed oxidative stress as a key contributor to the pathogenesis of BPH [17–20]. Moreover, compensatory cellular proliferation may be triggered by oxidative stress, which eventually leads to the growth of hyperplastic prostate tissue, whereas the factors that induce a more oxidative state in the prostate remain unclear.

The effect of experimental periodontitis on prostatic hyperplasia has not yet been reported. Under the framework of the hypothetical oral-prostate axis, the present study hypothesized that enhanced oxidative damage and inflammation might contribute to the aggravated pathogenesis of BPH by periodontitis. Herein, we established a rat model of ligature-induced periodontitis and testosterone-induced BPH to explore the possible relationship between periodontitis and BPH development. We also conducted an *in vitro* experiment on *Porphyromonas gingivalis* lipopolysaccharide- (LPS-) induced BPH-1 cells to determine whether oxidative stress is involved in this relationship, thus providing certain experimental evidence for the association of periodontitis with BPH and clarifying the potential mechanism linking the two diseases.

## 2. Materials and Methods

### 2.1. Animals

Male adult Sprague-Dawley (SD) rats weighting 300-350 g were obtained from the Animal Experiment Center of Zhongnan Hospital of Wuhan University and acclimated (temperature-controlled room on a half-day light/dark cycle with free access to water and food) for 1 week. All procedures in handling animals were adhered to the guidelines of the Institutional Animal Care and Use Committee (IACUC) of Wuhan University (IACUC animal approval protocol #2018119).

### 2.2. Experimental Design

The rats were randomly divided into four groups (*n* = 5/group): (1) a sham-operated group (control) undergoing sham operation for castration and subcutaneous injection of 0.9% saline solution (5 mg/kg/day) for four weeks, (2) a testosterone-induced BPH group (BPH) undergoing castration and subcutaneous injection of testosterone propionate (5 mg/kg/day) (Ningbo Second Hormone Factory, Ningbo, China) for four weeks [21], (3) a ligature-induced experimental periodontitis group (EP) undergoing ligation of sterile nylon thread around the cervical of bilateral maxillary first and second molars [22] and subcutaneous injection of 0.9% saline solution (5 mg/kg/day) for four weeks, and (4) a composite group (EP+BPH) undergoing castration and subcutaneous injection of testosterone propionate as the testosterone-induced BPH group; simultaneously, the maxillary first and second molars of rats were treated the same way as those of the ligature-induced EP group. The above surgical procedures were conducted under anesthesia by intraperitoneal injection of sodium pentobarbital (40 mg/kg), and all rats received subcutaneous injections in a week after the surgeries.

### 2.3. Harvest of the Rat Prostate

After 4 weeks of the injection administration, all rats were euthanized using an overdose of anesthetic. Prostatic ventral lobes and seminal vesicles were harvested, and the wet weight of the isolated prostate was measured immediately. Portions of the ventral prostate were kept in 4% paraformaldehyde (Dalian Meilun Biotechnology Co., Ltd., Dalian, China) for histological and immunohistochemical analyses. The remaining prostate tissues were frozen in liquid nitrogen for subsequent molecular analyses.

### 2.4. Microcomputed Tomographic (Micro-CT) Analyses of Alveolar Bone

Bilateral maxillary alveolar bone-contained molars were harvested and fixed with 4% paraformaldehyde. The right maxillae were dissected free of soft tissues to evaluate alveolar bone loss in each group by micro-CT (Skyscan 1176, Bruker, Kontich, Belgium). The X-ray generator was operated at a source voltage of 58 kV and source current of 431 *μ*A with an exposure time of 1000 ms and an image pixel size of 9 *μ*m. Three-dimensional (3D) reconstruction was performed by the software NReCon (Bruker, Kontich, Belgium) after scanning. 3D images of alveolar bones were obtained by the software CTvox (Bruker, Kontich, Belgium). The cementoenamel junction to alveolar bone crest (CEJ-ABC) was measured by DataViewer 1.5.2.4 (Bruker, Kontich, Belgium) for the maxillary second molar of four sites as follows: the proximal buccal, proximal palatal, distal buccal, and distal palatal. The CEJ-ABC distance was then calculated for statistical analysis. The residual left side of the maxillae was subsequently used for histological evaluation.

### 2.5. Histopathological Analyses

The fixed prostate tissues and periodontal tissues were embedded into paraffin after being dehydrated in gradient alcohol for dehydration. And then, 4 *μ*m sections were prepared with a microtome (Leica Biosystems, Shanghai, China) for histological examinations. The H&E staining was conducted according to standard procedures, and images were obtained with a light microscope (Leica DFC295, Wetzlar, Germany).

Masson's trichrome staining was applied for the obtained prostate paraffin sections (4 *μ*m) to highlight the microstructures of prostatic epithelia, smooth muscle (SM) cells, and collagen fibers (CF) after being stained red, dark red, and blue, respectively. Histological alterations of prostate tissues were observed by inverted phase contrast microscope (Cat. #DMi1, Leica, Wetzlar, Germany). The epithelial thickness of ventral prostate tissues and area percentages of epithelia, SM, and CF were quantified then analyzed by ImageJ software (ImageJ, National Institutes of Health, USA).

### 2.6. Immunohistochemistry Staining for Ki67

Tissue sections (4 *μ*m) were prepared for immunohistochemical study. The sections were processed with deparaffinization, retrieval in EDTA solution (Aspen, Wuhan, China), and incubation in 3% hydrogen peroxide (Sinopharm Chemical Reagent Co., Ltd., Shanghai, China). The samples were incubated overnight at 4°C with primary antibody of rabbit polyclonal anti-Ki67(Affinity Biosciences, Cincinnati, USA), then incubated with the HRP-labeled goat anti-rabbit second antibody (Aspen, Wuhan, China) at 37°C for 50 min. Brown-stained nuclei in cells were considered positive and the Ki67-positive rate was quantified by ImageJ software.

### 2.7. Terminal Deoxynucleotidyl Transferase-Mediated dUTP Nick End Labeling Assay

The determination of prostate cell apoptosis was evaluated by terminal deoxynucleotidyl transferase- (TdT-) mediated deoxyuridine triphosphate (dUTP) nick end labeling (TUNEL) assay according to the manufacturer's protocol. The deparaffinized prostate sections (4 *μ*m) were digested with proteinase K (Roche molecular biochemical kit, Germany) and incubated in permeabilization buffer (Aspen, Wuhan, China). The tissues were further processed with the TUNEL reaction mixture (TdT and dUTP) and DAPI and finally were sealed by antifade fluorescence mounting medium (Aspen, Wuhan, China). The images of immunofluorescence staining were obtained with tissue cell nuclei being stained blue and TUNEL-positive nuclei stained green. Positive staining area and cell numbers were analyzed by ImageJ software, and the apoptosis rate (%) was estimated as the (number of positive cells/the total number of epithelial cells) × 100.

### 2.8. Western Blot Analysis for Bax and Bcl-2 Protein Expression

Prostatic tissues were homogenized using RIPA protein lysis buffer (Beyotime Biotechnology, Shanghai, China) in an ice bath. The supernatant of protein solution was collected after centrifugation (13,300 rpm for 30 min) at 4°C. Bicinchoninic acid (BCA) protein assay kit (Biosharp, Shanghai, China) was used to determine the protein concentrations of the samples. Western blot was performed with 10% sodium dodecyl sulfate-polyacrylamide gel electrophoresis (SDS-PAGE), and protein samples were separated by SDS-PAGE then transferred to the polyvinylidene fluoride (PVDF) membrane (Millipore, Billerica, MA, USA). The membranes were blocked in 2% BSA for 1 h then incubated with the rabbit monoclonal anti-Bax primary antibody at 1 : 1000 (Abcam, Cambridge, USA) or rabbit polyclonal anti-Bcl-2 primary antibody at 1 : 1000 (Abcam, Cambridge, USA) at 4°C overnight. Then, membranes were incubated with HRP-conjugated goat anti-rabbit second antibody at 1 : 5000 (Boster, Wuhan, China) at room temperature for 1 h after washing. GAPDH (Abcam, Cambridge, USA) was used as a loading control. Thereafter, immunodetection bands were reacted with an Enhanced Chemiluminescence (ECL) kit (Beyotime Biotechnology, Shanghai, China) and analyzed with an Alliance Q9 Chemiluminescence Imager (Uvitec, UK). The list of antibodies used for western blot analysis is presented in Table 1.

### 2.9. Determination of Inflammatory Cytokines

Blood samples were collected from an abdominal aorta before the rats were sacrificed, and plasma was separated by centrifugation (3000 rpm for 15 min) at 4°C. Plasma samples were analyzed for tumor necrosis factor-*α* (TNF-*α*), interleukin-6 (IL-6), interleukin-1*β* (IL-1*β*), and C-reaction protein (CRP) using ELISA kits (ELK Biotechnology, Wuhan, China) according to the manufacturer's instructions.

### 2.10. Determination of Oxidative Stress Markers

#### 2.10.1. Human Prostatic Cell Line

Human benign prostatic enlargement epithelial cell line BPH-1 was obtained from the Department of Urology in Zhongnan Hospital of Wuhan University and cultured as previously described [23].

#### 2.10.2. Determination of ROS

The production of ROS induced by *Porphyromonas gingivalis* LPS was evaluated following the ROS assay kit (Dojindo, Kumamoto, Japan) manual. Briefly, 1 × 10^5^ BPH-1 cells/well were seeded into 6-well plates with RPMI-1640 (Hyclone, USA), containing 10% fetal bovine serum (Hyclone, USA), and cultured at 37°C for 24 h. The medium was replaced with RPMI-1640 containing 1 *μ*g/mL *Porphyromonas gingivalis* LPS (Sigma, SMB00610) and cultured at 37°C for a further 24 h. The supernatant was removed, and highly sensitive DCFH-DA dye working solution (Dojindo, Kumamoto, Japan) was added then incubated at 37°C for 30 min. The changes in the levels of ROS were detected using flow cytometry.

#### 2.10.3. Determination of H_2_O_2_

The concentration of H_2_O_2_ induced by *Porphyromonas gingivalis* LPS was evaluated using the H_2_O_2_ assay kit (Beyotime Biotechnology, Shanghai, China). BPH-1 cells were treated with 1 *μ*g/mL *Porphyromonas gingivalis* LPS for 24 h as above and collected into a centrifuge tube, then H_2_O_2_ lysis was added for homogenization of cells. The supernatant was collected after centrifuging at 12000 g for 5 min at 4°C. Then, a 50 *μ*L sample or standards and a 100 *μ*L hydrogen peroxide detection reagent were added and incubated at room temperature for 30 min. The changes in the levels of H_2_O_2_ were detected using a microplate reader (Thermo Scientific Varioskan Flash).

### 2.11. Statistical Analysis

The data were expressed as the means ± standard error of mean (SEM). Statistical analysis was performed using SPSS 17.0 software (SPSS, Inc., Chicago, IL, USA). The differences between groups were analyzed with an independent-sample test or one-way analysis of variance (ANOVA); Bonferroni correction was applied for post hoc comparisons. *p* < 0.05 was considered statistically significant.

## 3. Results

### 3.1. Micro-CT and Histopathological Analyses of Alveolar Bone

Experimental periodontitis was established in the EP model and EP+BPH model, which was confirmed by the analyses of micro-CT. The 3D images provided the clear morphology views of the maxillary alveolar bones from different angles (Figure 1(a)), which showed obvious bone resorption, especially for the residual ridge between the first molar and the second molar. Statistical analysis also demonstrated that the CEJ-ABC of the animals in EP and EP+BPH was significantly increased when compared with the control and BPH groups (control vs. EP/EP+BPH: *p* < 0.01; BPH vs. EP/EP+BPH: *p* < 0.01) (Figure 1(b)). Our results indicated that all rats from the EP and EP+BPH groups were successfully induced to the ligature-induced experimental periodontitis. Periodontal histopathologic analysis of the regions of the second molar showed the structures of gingiva, periodontal ligament, alveolar bone, and cementum. The rats suffered experimental periodontitis (EP and EP+BPH groups) and observed the erosion of gingival epithelium with infiltrated inflammatory cell, derangement of collagen fiber within the periodontal ligament, loss of epithelial attachment, and breakdown of alveolar bone (Figure 1(c)). And no obvious pathological change was found between the BPH group and the control group.

### 3.2. Effects of Experimental Periodontitis on the Histological Alteration of Prostate Tissues

#### 3.2.1. Prostate Weight and Index

All the rats undergoing castration and induced testosterone showed a significant increase in prostate volume. Prostate enlargement in rats can be induced in testosterone-treated rats, which was aggravated by periodontal ligation (Figure 2(a)). Prostate weight and index were significantly enhanced by 66% and 80% in testosterone treated rats, respectively, when compared to the control group. Simultaneous periodontitis caused an obvious increase in the prostate weight by 59% and the prostate index by 81%, respectively, when compared to the control group (Figure 2(b)). Body weight was measured before the experiments and after the 4-week injection. At the end of the experiment, rats in the composite group showed the lowest body weight, followed by those in the BPH and EP groups (Table 2).

#### 3.2.2. Histopathological Examination of Ventral Prostate Tissues

Microscopic examination (H&E staining) showed that prostatic tissues obtained from control rats remain as a normal structure with numerous acini containing homogenous acidophilic material (Figure 2(c)), whereas prostates taken from rats injected with testosterone displayed marked glandular hyperplasia and a decreased glandular luminal area compared to the control animals (Figure 2(c)). Masson's trichrome staining showed that testosterone-treated rats displayed increased stromal cells in the prostate (Figure 2(d)). Quantitative analysis of histological components suggested that the EP group presented with a significantly thickened epithelium; the BPH group showed increased epithelium, SM, and CF; and the EP+BPH group demonstrated the most obvious increasing of hyperplasia of epithelia, SM, and CF, with all *p* < 0.05 (Figures 2(e) and 2(f)).

### 3.3. Effects of Experimental Periodontitis on the Proliferation and Apoptosis of Prostate Tissues

#### 3.3.1. Immunohistochemical Detection of Ki67

The proliferation marker Ki67 protein expression was evaluated immunohistochemically and showed 8.80% positive rate in the control group (Figure 3(a)). However, in the group which received periodontal ligation or testosterone alone, an increment of stained cells was noted (approximately 14.01% and 17.08%), suggesting an elevation of the proliferation rate (Figures 3(b) and 3(c)). Simultaneous periodontitis and BPH further increased the number of Ki67-positive cells (Figure 3(d)), in comparison to the BPH rats. The quantitative analysis results (Figure 3(e)) indicated that the Ki67-positive rate was significantly higher in the experimental groups than in the control, among which the EP+BPH group was at the highest degree of proliferation. In addition, significant differences were detected between the groups (all *p* < 0.01).

#### 3.3.2. Determination of Apoptosis of Prostate Tissue

TUNEL assay showed obvious characteristic of antiapoptosis of prostate cells in the testosterone-treated rats (Figures 4(a)–4(d)). The quantitative analysis also revealed a significant decrease of the apoptosis rate in BPH and EP+BPH groups (Figure 4(e)). The protein expression levels of Bax and Bcl-2 were also detected to investigate the cell apoptosis of the rat prostate (Figure 4(f)). The apoptosis inducer Bax was shown to be downregulated and the apoptosis inhibitor Bcl-2 upregulated in the experimental groups compared with the control (Figures 4(g) and 4(h)), which was obviously observed in the composite group, which further confirmed the explained antiapoptosis of prostate cells in testosterone-treated rats.

### 3.4. Effects of Experimental Periodontitis on Plasma Levels of Inflammation Cytokines in BPH Rats

Periodontitis and BPH both significantly enhanced inflammatory marker levels of TNF-*α*, IL-6, IL-1*β*, and CRP in plasma when compared to the control group. Simultaneous periodontitis and BPH synergistically further enhanced inflammation cytokine levels than when treated alone (Figure 5), which indicate a potential effect of experimental periodontitis on systemic inflammation levels in BPH rats.

### 3.5. Effects of Porphyromonas gingivalis LPS on the Generation of ROS and H_2_O_2_ in BPH-1 Cells

Our results showed that *Porphyromonas gingivalis* LPS increased the intracellular levels of ROS in BPH-1 cells after 24 h of exposure (Figures 6(a) and 6(b)), with significant difference from the untreated group (Figure 6(c)). In line with the enhanced generation of ROS, the concentration of H_2_O_2_ also significantly increased after *Porphyromonas gingivalis* LPS exposure for 24 h (Figure 6(d)).

## 4. Discussion

The high prevalence of BPH in patients with periodontitis has become a major worldwide health problem affecting elderly male populations. Thus, it is quite crucial to clarify the mechanism accounting for the aggravation of BPH by periodontitis. In this study, for the first time, we established rat models to examine the effect of experimental periodontitis on prostatic hyperplasia, which provide the evidence that periodontitis may promote the development of BPH through the regulation of oxidative stress and systemic inflammation.

In previous animal studies, it was proven that injection of testosterone is an established model for induction of BPH in rats [21], and periodontal ligation is an established model for induction of periodontitis in rats [22]. To our knowledge, this is the first study examining the potential role of periodontitis in the development of prostatic hyperplasia based on animal models. In our study, comparison models were successfully constructed and verified by histopathological findings. Testosterone-induced hyperplasia indicated a significant increase in prostate weight and prostate index. Periodontitis significantly promoted testosterone-induced hyperplasia which was indicated by the aggravation of the pathological structure alterations in the composite model. Histologically, the observation of pathology changes in testosterone-treated groups, especially in EP+BPH, indicated a predisposition to BPH and an aggravated effect of periodontitis on prostate hyperplasia. The imbalance of cell proliferation and apoptosis is known to be involved in the development of BPH [24]. Furthermore, the Bax/Bcl-2 ratio has been widely studied as an influential factor for progression of apoptosis in developing BPH [25]. This is consistent with our results, as experimental groups present increased Ki67 expression and decreased apoptosis of prostate cells. Additionally, our study found a downregulated Bax and upregulated Bcl-2 expression in the experimental groups, in which the most obvious changes were detected in the EP+BPH group, which is consistent with the manifestations of BPH [26, 27] and further defined the effect of periodontitis on the apoptosis of prostate tissues.

Accumulated research has confirmed the inflammatory association between periodontitis and BPH based on epidemiological investigation or clinical data, which probably occurs through dissemination of proinflammatory cytokines that can further exaggerate the preexisting inflammation [28, 29]. Experimentally, numerous researches have confirmed inflammation as one of the factors by which testosterone can induce BPH [30, 31]. In this study, the markedly raised inflammatory cytokines of IL-6, IL-1*β*, TNF-*α*, and CRP in testosterone-induced models could support the hypothesis. Also, the role of oxidative stress was highlighted in testosterone-induced BPH [32]. Testosterone has been reported to increase prostatic cellular metabolism, thus inducing a wide production of free radicals in combination with dampening the antioxidant system, leading to cell dysfunction [33]. Our data found that LPS from *Porphyromonas gingivalis* induced a significantly higher level of intracellular ROS and H_2_O_2_ in BPH-1 cells, indicating oxidative stress might provide a molecular link between periodontal disease and BPH development.

Oxidative stress and inflammation underpin several age-related diseases, and their mechanisms are inextricably linked. For instance, oxidative stress may increase the production of proinflammatory cytokines thus triggering systematic inflammation [34]. Anti-inflammatory cascades are linked to decreased oxidation, both playing key roles in cellular and tissue damage, influencing the development of multiple age-related diseases [35, 36]. Inflammation and oxidative stress significantly contribute to prostatic remodeling. Although the factors that produce a more oxidative state in the prostate remain unclear, studies indicated that the hormonal environment (i.e., testosterone) and chronic inflammation might be relevant in this process [37]. Indeed, the onset of prostatic tissue inflammation and oxidative stress imbalance can result in the accumulation of inflammatory cytokines and other growth factors [38]. This is in line with our noticed increase in the plasma levels of inflammatory cytokines in testosterone-treated rats. Furthermore, it is consistent with their famous role in promoting prostate cell proliferation.

## 5. Conclusions

In conclusion, our findings demonstrate that periodontitis might promote BPH development through regulation of oxidative stress and inflammatory process. The present study brings early evidence to this field; however, more studies should be done to clarify the role of these specific bacteria and their potential to be exploited as new biomarkers for BPH. This may help to reveal new strategies to combat BPH.

## Figures and Tables

**Figure 1:** Alveolar bone loss and histological changes in rat periodontal tissues. (a) Representative images obtained by micro-CT, including the surface of the bone, the trabecular structure inside, the regain of root furcation of the second molar, and the bone surrounding the roots. The red lines showed the linear distance from the cementoenamel junction (CEJ) to the alveolar bone crest (ABC) for the maxillary second molar. (b) Quantitative analysis of the CEJ-ABC distance from the control, EP, BPH, and EP+BPH groups. Data are presented as mean ± SEM (^∗∗^*p* < 0.01). (c) Representative figures from HE staining for the second maxillary alveolar bones (arrows indicate inflammatory changes in the gingival epithelium, scale plates indicate linear distance from CEJ to ABC). Scale bar = 500 *μ*m; original magnification ×40.

**Figure 2:** Typical photographs and histological examination of rat prostate tissues. (a) Photographs of (1) ventral prostate, (2) bladder, and (3) seminal vesicle from the control, EP, BPH, and EP+BPH groups. (b) A bar graph for prostate weight index (prostate weight of each animal/body weight of each animal) × 1000. (c) Representative figures from H&E staining for the prostate tissues. (d) Representative figures from Masson's trichrome staining for the prostate tissues. Prostatic epithelial cells, smooth muscle (SM) cells, and collagen fibers (CF) were stained red, dark red, and blue, respectively. Scale bar = 200 *μ*m; original magnification ×200. (e) A bar graph for epithelial thickness of ventral prostate tissues. (f) A bar graph for area percentage of different components (epithelia, SM, and CF) from the control, EP, BPH, and EP+BPH groups. Data are presented as mean ± SEM (^∗^*p* < 0.05, ^∗∗^*p* < 0.01, and ^∗∗∗^*p* < 0.001).

**Figure 3:** Ki67 staining for detecting cell proliferation of prostate tissues. (a–d) Representative figures from Ki67 immunohistochemical staining for ventral prostates of the control, EP, BPH, and EP+BPH groups, respectively. Scale bar = 200 *μ*m; original magnification ×400. (e) A bar graph for rate (%) of Ki67-positive cells in rat prostate. Data are presented as mean ± SEM (^∗∗^*p* < 0.01).

**Figure 4:** Terminal deoxynucleotidyl transferase-mediated dUTP nick end labeling (TUNEL) assay and western blot analysis for detecting cell apoptosis of prostate tissues. (a–d) Representative figures from TUNEL staining of prostate tissues for the control, EP, BPH, and EP+BPH groups, respectively. Tissue cell nuclei were stained blue with DAPI; TUNEL-positive nuclei were stained green. Scale bar = 200 *μ*m; original magnification ×200. (e) A bar graph for apoptosis rate (%) of TUNEL-positive cells in rat prostate. (f) Representative protein bands for Bax and Bcl-2 in prostate tissues among the indicated groups. (g) Quantitative analysis of the protein level of Bax relative to GAPDH. (h) Quantitative analysis of the protein level of Bcl-2 relative to GAPDH. Data are presented as mean ± SEM (^∗^*p* < 0.05, ^∗∗^*p* < 0.01, and ^∗∗∗^*p* < 0.001).

**Figure 5:** Enzyme-linked immunosorbent assay (ELISA) for detecting the inflammatory cytokine levels of (a) TNF-*α*, (b) IL-6, (c) IL-1*β*, and (d) CRP in plasma of rats. TNF-*α*: tumor necrosis factor-*α*; IL: interleukin; CRP: C-reaction protein. Data are presented as mean ± SEM (^∗^*p* < 0.05, and ^∗∗^*p* < 0.01).

**Figure 6:** Assessment of intracellular ROS and H_2_O_2_ production in BPH-1 cells treated with *Porphyromonas gingivalis* LPS. The effect of *Porphyromonas gingivalis* LPS on the production of ROS was evaluated by flow cytometry in BPH-1 cells, either (a) untreated control or (b) *Porphyromonas gingivalis* LPS exposure for 24 h. (c) A bar graph for intracellular level of ROS (%) in BPH-1 cells, either untreated (BPH) or treated with *Porphyromonas gingivalis* LPS for 24 h (LPS-BPH). (d) A bar graph for intracellular expression of H_2_O_2_ in BPH-1 cells, either untreated (BPH) or treated with *Porphyromonas gingivalis* LPS for 24 h (LPS-BPH). ROS: reactive oxygen species; H_2_O_2_: hydrogen peroxide. Data are presented as mean ± SEM (^∗^*p* < 0.05, and ^∗∗^*p* < 0.01).

**Table 1:** List of antibodies used for western blot analysis.

Primary antibodies	Source species	Antibody supplier	Dilution buffer	Dilution ratio	Dilution buffer supplier
GAPDH	Rabbit	Abcam, ab181602	QuickBlock™ Primary Antibody Dilution Buffer	1 : 1000	Beyotime, P0256
Bax	Rabbit	Abcam, ab182733	QuickBlock™ Primary Antibody Dilution Buffer	1 : 1000	Beyotime, P0256
Bcl-2	Rabbit	Abcam, ab196495	QuickBlock™ Primary Antibody Dilution Buffer	1 : 1000	Beyotime, P0256
Secondary antibody					
HRP-goat anti-rabbit		Boster, BA1054	1 × TBST	1 : 5000	Solarbio, T1081

**Table 2:** Variation of physiological parameters in rat models.

Group	Body weight (g)		Prostate weight (mg)	Prostate weight index (×10^3^)
	Initial	Final		
Control	304.60 ± 5.99	424.60 ± 12.36	609.00 ± 23.18	1.44 ± 0.08
EP	298.20 ± 4.22	412.20 ± 9.09	613.20 ± 32.16	1.49 ± 0.06
BPH	306.00 ± 15.21	393.80 ± 21.04	1009.4 ± 26.10^∗∗∗^	2.59 ± 0.14^∗∗∗^
EP+BPH	298.00 ± 8.44	370.40 ± 5.22	969.0 ± 61.01^∗∗∗^	2.61 ± 0.13^∗∗∗^

Prostate weight index = (prostate weight of each animal/body weight of each animal) × 1000. Data are presented as mean ± SEM. ^∗∗∗^*p* < 0.001 vs. control rats; ^∗∗∗^*p* < 0.001 vs. EP rats.

## Data Availability

The data used to support the findings of this study are included within the article.
